# A High-Precision Classification Method of Mammary Cancer Based on Improved DenseNet Driven by an Attention Mechanism

**DOI:** 10.1155/2022/8585036

**Published:** 2022-05-14

**Authors:** Xuebin Xu, Meijuan An, Jiada Zhang, Wei Liu, Longbin Lu

**Affiliations:** ^1^School of Computer Science and Technology, Xi'an University of Posts & Telecommunications, Xi'an Shaanxi 710121, China; ^2^Shaanxi Key Laboratory of Network Data ANalysis and Intelligent Processing, Xi'an University of Posts & Telecommunications, Xi'an Shaanxi 710121, China

## Abstract

Cancer is one of the major causes of human disease and death worldwide, and mammary cancer is one of the most common cancer types among women today. In this paper, we used the deep learning method to conduct a preliminary experiment on Breast Cancer Histopathological Database (BreakHis); BreakHis is an open dataset. We propose a high-precision classification method of mammary based on an improved convolutional neural network on the BreakHis dataset. We proposed three different MFSCNET models according to the different insertion positions and the number of SE modules, respectively, MFSCNet A, MFSCNet B, and MFSCNet C. We carried out experiments on the BreakHis dataset. Through experimental comparison, especially, the MFSCNet A network model has obtained the best performance in the high-precision classification experiments of mammary cancer. The accuracy of dichotomy was 99.05% to 99.89%. The accuracy of multiclass classification ranges from 94.36% to approximately 98.41%.Therefore, it is proved that MFSCNet can accurately classify the mammary histological images and has a great application prospect in predicting the degree of tumor. Code will be made available on http://github.com/xiaoan-maker/MFSCNet.

## 1. Introduction

Cancer is one of the major killers threatening human health and life [1], among which mammary cancer is the most common cancer among women. According to the data released by the International Center for Research on Cancer (IARC), a subordinate of the World Health Organization (WHO) in 2012, mammary cancer [2] is the second leading cause of death among women, and its incidence is on the rise year by year and the trend of younger. Since the late 1970s, the incidence of mammary cancer has been on the rise worldwide. The incidence of mammary cancer in China is increasing at a rate of 3 to 4 percent year, and the five-year survival rate is 73%. In Americans, more than 80% of Americans are diagnosed with mammary cancer at stage I. In China, the probability of diagnosis of mammary cancer in I stage is less than 20%, and once detected, most of them have metastasized or spread. Therefore, for the treatment of mammary cancer, early diagnosis is particularly important. Delay in diagnosis is one of the main reasons for the high mortality rate from mammary cancer.

According to tumor property, mammary cancer can divide into benign tumor and malignant tumor. According to the specific category of mammary tumors, it can also divide into adenopathy, tubular adenoma, fibrous adenoma, phyllodes tumor, ductal cancer, lobular cancer, mucous cancer, papillary cancer, and other specific category; accurate diagnosis is an important basis for making corresponding treatment plan. Diagnosis of mammary cancer usually adopts radiological image analysis for preliminary examination, such as X-rays [3], ultrasound (B-ultrasound) [4], and thermal imaging [5], to determine abnormal sites. Then, if the test shows the possibility of malignant tissue growth, a mammary biopsy is performed. Biopsy, in which the tissue is taken and examined under a microscope for the presence or absence of cancer, is the only reliable method to identify a site as cancerous [6]. However, the traditional manual diagnosis requires experts with professional knowledge to carry out high-intensity work. Using computer-aided diagnosis (CAD), the automatic and accurate classification of mammary histological images can not only provide doctors with objective and accurate diagnosis reference but also improve the efficiency and accuracy of diagnosis.

Considering that DenseNet is a densely connected network, and DenseNet is directly connected to feature maps from different layers, this can fully combine the contextual information of pathological images, facilitate complex breast pathological image classification, enable feature reuse, and improve model efficiency. So in our paper, we focus on the problems of the existing research methods of pathological image classification; using the design ideas of DenseNet and SENet, a high-precision classification model of mammary historiography image is proposed, which integrates spatial and channel feature information. DenseNet only realizes spatial feature fusion, while the innovation of SENet lies in the addition of SE module, so that the network can learn the relationship between channels and the importance degree of features of different channels. Using the thought of SENet, under compression and motivation into DenseNet operation, the features of the network can not only realize space fusion but also can learn the relationship between the characteristics of the channel, to further improve the performance of network. The network model was named classification of mammary cancer fusing spatial and channel features network (MFSCNet). Moreover, by using data preprocessing and data enhancement to process the dataset, model training and testing are conducted on the Breast Cancer Histopathological Database (BreakHis), which verifies that the proposed algorithm can carry out high-precision classification of mammary histopathological images.

## 2. Related Work

It is difficult to classify the pathological images of mammary cancer because of the slight difference between the pathological images and the overlap between cells, and most studies are based on small self-made dataset and have not been published, making it difficult to replicate existing results for comparison. But still, experts and scholars have carried out researches on the classification of pathological images and achieved good results. The research methods can be divided into two categories.

One is to use feature descriptors and machine learning algorithms to classify anthologize image of mammary. Feature descriptors are used to extract image morphology, texture, and other relevant feature information, and then, a machine learning classifier is used to classify them, so as to realize the classification of anthologize image of mammary [7, 8]. Zhang et al. [9] proposed a classification scheme based on the kernel principal component analysis (KPCA) model to classify mammary cancer histopathology images into benign and malignant, with an accuracy of 92%. This method uses a simple dataset that covers only the important areas of the pathological images, so it has a high accuracy. However, it is often difficult to find the region of interest that contains only the most important tissue in a biopsy scan. Spanhol et al. [10] introduced a Breast Cancer Histopathological Database (BreakHis) in the literature, on which different feature descriptors and different traditional machine learning classification algorithms were used to classify cases as benign or malignant, with an accuracy range of 80% to 85%. Chan and Tuszynski [11] used SVM to classify mammary cancer anthologize images at 40x magnification and classified mammary tumors into 8 subtypes (multiclass classification) with an accuracy rate of only 55.6%. Visible feature descriptors and machine learning algorithms cannot achieve high-precision classification of mammary cancer pathological images, especially multiclass classification of mammary subtypes. Irfan et al. [12] use pixel-level semantic segmentation of ultrasound mammary lesions with dilation factors and a mask-based ultrasound imaging dataset. After the segmentation stage, compared to the ground truth mask, erosion and size filters are performed on the extracted lesions, to remove noise in segmented lesions. And for transfer learning features, the DenseNet201 deep network is used, and for feature activation, the proposed CNN is used. Single eigenvectors and fusion-based eigenvectors were validated on both validation techniques using the SVM classifier variant, with greater improvement in correctly identifying true positives. The fusion version of the final feature vector and SVM outperforms other algorithms with an accuracy rate of 98.9%. Zebari et al. [13] propose a hybrid threshold method and machine learning method to extract the region of interest in mammograms; exported ROI is divided into five distinct blocks. Using wavelet transform to capture high and low frequencies in different subbands, noise suppression is performed on each resulting block. An improved fractal dimension (FD) approach is proposed, called multi-FD (M-FD), is proposed to extract multiple features from each denoised block. Then, the number of feature extractions is reduced by a genetic algorithm, and 5 classifiers are trained and together with an artificial neural network (ANN) to classify the features extracted from each block. Finally, the results of the 5 blocks are fused to obtain the final decision. The method was tested and evaluated on four mammography datasets, MIAS, DDSM, INbreast, and BCDR. The proposed method yields better results on the INbreast dataset in the single-dataset evaluation, on the remaining datasets in the dual-dataset evaluation.

The other is the classification algorithm based on deep learning, which uses the network structure with the convolution layer as the core to achieve a more effective feature learning process, so it has better performance than the traditional machine learning classification algorithm. By continuously automatically optimizing the classification loss function, useful features can be learned directly from the input original images, so as to realize the classification of mammary histological images. Region of interest of pathological image is avoided, and the classification accuracy is improved. In 2016, Spanhol et al. [14] used a deep constructional neural network (DCNN) model AlexNet to classify the benign and malignant pathological images of mammary cancer, with an accuracy of 85% ~90%. It is significantly higher than the machine learning method used in literature. Zhan et al. [15] proposed a classification method for mammary pathology images based on the deep constructional neural network based on Inception V3 and improved it; average accuracy of the binary classification experiment was 97%, but only 89% in the multiclass classification experiment. Wei et al. [16] proposed a data enhancement method and a new CNN-based mammary cancer histopathological image classification method based on deep constructional neural networks (BICNN), and the accuracy of dichotomy reached 97%. Jiang et al. [17] proposed a small SE-ResNet module and a new learning rate scheduler. A mammary cancer histopathology image classification network (BHCNet) is designed. The experimental results show that the proposed method has a good classification performance. The accuracy of binary classification was 98.87% ~99.34%, and the accuracy of multi-class classification was 90.66% ~93.81%. In 2021, Lahoura et al. [18] propose a mammary cancer diagnosis framework based on cloud computing using extreme learning machine (ELM) as a classifier. They performed mammary cancer diagnosis on the WBCD dataset. Cloud computing can provide uninterrupted services anytime, anywhere and access the system at any time and also provided to improve the overall classification accuracy of the proposed model, and ELM does not need to adjust parameters such as weights and biases, making the classification algorithm faster and simpler. The experimental results of this method on the Wisconsin Breast Cancer Diagnostic (WBCD) dataset show an accuracy of 0.9868.

The classification algorithm proposed in this paper is shown in Figure 1. The basic process is as follows: After data preprocessing, the dataset of mammary pathology image is divided into training data and test data. Then, the training data is enhanced to obtain new training data. Then, the obtained data is trained in MFSCNet, and finally, the test data is input into the trained MFSCNet for testing, to complete the classification of mammary pathological images.

### 2.1. The Dataset

The dataset used in this study was the BreakHis dataset [10], which contains images of microbiopsies of benign and malignant mammary tumors. BreakHis is the largest and most comprehensive dataset in the histopathological image dataset published at present, and it has a variety of magnification ratios and relatively high recognition difficulty. Therefore, the persuasiveness of experiments on this dataset is better than other datasets. The BreakHis dataset is derived from 82 anonymous patients (24 benign patients and 58 malignant patients) from the Brazilian Laboratory of Pathological Anatomy and Cytopathology (P&D), with a total of 7909 pathological images of mammary cancer and 8 mammary cancer subtypes. BreakHis is divided into benign and malignant tumors. The dataset currently contains four different subtypes of benign mammary tumors: adenoma, fibroadenoma, tubular adenoma, and lobular tumor and four malignancies (mammary cancer): ductal, lobular, mucinous,and papillary carcinomas, with four amplification factors : 40x, 100x, 200x, and 400x. The image is in PNG format, RGB three-channel, and 700 × 460 pixels.  Table 1 shows the specific distribution of benign and malignant tumor images with different magnifications.  Figure 2 shows the image sample with magnification for the BreakHis database.

### 2.2. Data Preprocessing and Data Enhancement

Data preprocessing can improve the accuracy of analysis results and shorten the calculation process. In the tissue image, preprocessing is the key step to remove different types of noise. At the same time, data preprocessing can simplify the data, improve the training speed of network model, and thus improve the reliability of feature extraction and recognition. In addition, the pathological image data in BreakHis dataset adopt different staining methods, which will bring color differences to the histopathological images; this is not a big hurdle for a trained pathologist, but it is a big problem for automated image processing, which can have a big impact on the final results. Therefore, it is necessary to perform data preprocessing on the original dataset, but directly performing grayscale processing on the original image will cause information loss to the pathological image. In this paper, the method proposed in literature [19] is used to normalize the dataset. The color normalization scheme is to perform accurate blemish separation on the source image and the target image by sparse regularization nonnegative matrix, and the structural information of the source image is unchanged. The histopathological images before and after color normalization are shown in Figure 3.

The small amount of data is an important reason for the overfitting [20] of the model in deep learning training, while convolutional neural networks (CNN) are invariant to translation, viewing angle, size, or illuminance (or a combination of the above). Data augmentation is the process of using the invariance of convolutional neural networks to expand datasets through operations such as translation, rotation, and flipping, so as to increase the number of training samples and avoid the problem of overfitting of CNN. Since the pathological images of mammary cancer are rotation-invariant, pathologists can easily analyze the pathological images of mammary cancer from different perspectives without any changes in diagnosis [21]. However, for CNN, it is a different image from the previous one, but its label is consistent. Therefore, the model generalization ability obtained through data augmentation training is stronger. Data augmentation with different rotation angles is shown in Figure 4.

## 3. The Proposed Method

### 3.1. Convolutional Neural Network

The convolutional neural network (CNN) is a deep learning model or multilayer perceptron similar to an artificial neural network, which is commonly used to analyze visual images. Studies have proved that CNN has achieved great success and has been widely used in the computer vision field, which is suitable for processing tasks such as image classification and image recognition.

The structure of a CNN mainly consists of several convolutional layers and pooling layers, followed by at least one fully connected layer. In the convolution layer, there are multiclass convolution kernels with trainable weights. By convolving the image with each convolution kernel and adding bias in the convolution layer, multiclass feature graphs are finally generated. In the convolution layer, there are multiclass convolution kernels with trainable weights. By convolving the image with each convolution kernel and adding bias in the convolution layer, multiclass feature graphs are finally generated.

Figure 5 shows the structure diagram of the famous convolutional neural network for handwritten character recognition:

### 3.2. Dense Neural Network

The dense connected convolutional neural network (DenseNet) is a network structure proposed by Huang et al. [22] in 2017, which has achieved the optimal results on multiclass image classification datasets. Previously used networks, such as the convolutional layer of AlexNet, tend to have large the characteristic dimension. The idea of this network is to connect multiclass convolutional layers with very small characteristic dimensions in a dense way. It is to connect the output of all previous convolutional layers together as the input of the next convolutional layer. In this way, using only *n* layers, *n* (*n* + 1)/2 connections can be obtained; thus, it fits more complex functions with fewer parameters. A group of such convolutional layers is called a Dense Block, and the characteristic dimension of each convolutional layer is called the growth rate. Among these modules, there is a convolution layer with a convolution kernel length and width of 1 and an average pooling layer with a kernel length and width and step size of 2.

DenseNet is essentially a convolutional neural network. The network consists of *L* layers, each of which performs a nonlinear transformation*H*_*i*_, where it is the index of the layer *l*, *H*_*l*_ could be the BN layer, ReLU activation functions, and the composition of pooled or convolutional layers. We define the input image as *x*_0_, and the output of layer *l* as *x*_*l*_.

In a traditional convolutional neural network, we take the output of layer *l* as the input of layer *l* + 1; the formula can be expressed as

(1) $$\begin{array}{c} x_{l}=H\left(x_{l-1}\right). \end{array}$$

In DenseNet, to further improve the flow of information between layers, a different connectivity pattern called dense connectivity is proposed, with the introduction of direct connections from any layer to all subsequent layers.  Figure 6 illustrates the DenseNet layout, layer *l* receives as input the feature graph of all previous layer *x*_0_, *x*_1_, ⋯, *x*_*l*−1_. The formula can be expressed as

(2) $$\begin{array}{c} x_{l}=H_{L}\left(\left[x_{0},x_{1},\cdots ,x_{l-1}\right]\right), \end{array}$$

where [*x*_0_, *x*_1_, ⋯, *x*_*l*−1_] means to stack the feature graph of *x*_0_, *x*_1_, ⋯, *x*_*l*−1_ on the channel dimension.

### 3.3. Squeeze and Excitation Network

To solve the problem that the traditional convolution does not utilize the feature map channel information, momenta's Hu et al. [23] propose a deep convolutional neural network squeeze-and-excitation network (SENet). The main innovation is the squeeze-and-excitation module. The two operations are compression and excitation. SENet is a very simple and efficient attention mechanism network model with low complexity and computational complexity. It is divided into squeeze and excitation parts L0. The basic network structure of SENet is shown in Figure 7. Its main processing process is as follows.

- Preprocessing: the original image is obtained through a series of CONV and pooling operations to obtain a CXHXW size feature map
- Squeeze processing: the feature map is compressed by global average pooling and get the feature map of size 1 × *l* × *C*. It is equivalent to compressing the original *H* × *W* dimension feature into *L* dimension, and the *I* dimension feature graph has the global receptive field of *H* × *W* dimension
- Excitation operation: a full connection layer is used to carry out nonlinear transformation on the feature map of 1∗1∗*C* to predict the importance of each channel, and then through the operation of ReLU and full connection, which is a gate mechanism similar to that in the cyclic neural network, two full connection layers are used to enhance nonlinearity and better fit the correlation between channels.

### 3.4. Pathological Image Classification of Mammary Cancer

The core idea of DenseNet is to establish connections between different layers to create a better network structure than ResNet, further reducing the gradient disappearance problem. Moreover, the network is very narrow, which greatly reduces the number of parameters and helps to suppress the overfitting problem. The reduction in the number of parameters also reduces the amount of calculation, which often appears in the small target detection scene. Compared with ResNet, DenseNet can achieve better results with fewer training parameters [22, 24]. Therefore, the basic network model used in this paper is DenseNet121 with a small number of training parameters, and the total number of training parameters is far less than ResNet18, DenseNet169, DenseNet201, etc. The comparison of the specific number of parameters is shown in Table 2. However, DenseNet only realizes spatial feature fusion, while the innovation of SENet lies in the addition of the SE module, so that the network can learn the relationship between channels and the importance degree of features of different channels. And in our paper, optimization operations such as local pooling, global pooling, and variance were added to the compression operation of SENet. The optimized structure of SENet is shown in Figure 8. Then, pruning was carried out in DenseNet, which resulted in fewer parameters and shorter training time, which got even better results.

The thought of this article and SENet, under compression and motivation into DenseNet121 operation, this paper proposes a blend of the space characteristics and channel characteristic of network (MFSCNet) mammary cancer pathology image classification; the features of the network can not only realize space fusion but also can learn the relationship between the characteristics of the channel, to further improve the performance of network. Depending on the amount of insert position and insertion of the SE module, the design of the three different MFSCNet network models, respectively, MFSCNet A, MFSCNet B, and MFSCNet C, and through the experimental analysis to find out about the highest mammary tissue pathological image classification accuracy. The SE module is inserted as shown in Figure 9.

## 4. Experimental Results and Analysis

### 4.1. Evaluation Metrics

The classification results are reported and evaluated through two assessment methods. One is the purpose of this experiment is to classify mammary histopathological images; the evaluation indexes used include accuracy, precision, recall, and *F*1 score. The accuracy can be expressed by

(3) $$\begin{array}{c} \text{Accuracy}=\frac{\text{TP}+\text{TN}}{\text{TP}+\text{FP}+\text{TN}+\text{FN}}. \end{array}$$

TP (true positive) represents true cases, namely, the number of correctly predicted positive cases. Fn (false negative) represents the number of false negative cases that are wrongly predicted. FP (false positive) represents the number of false positive cases, that is, the number of wrongly predicted negative cases. TN (true negative) represents true negative cases, i.e., cases that are correctly predicted to be negative cases. The calculation formula of precision is as follows:

(4) $$\begin{array}{c} \text{Precision}=\frac{\text{TP}}{\text{TP}+\text{FP}}. \end{array}$$

The calculation formula of recall rate is as follows:

(5) $$\begin{array}{c} \text{Recall}=\frac{\text{TP}}{\text{TP}+\text{FN}}. \end{array}$$

The formula for calculating the *F*1 value is as follows:

(6) $$\begin{array}{c} F1=\frac{2*\text{Precision}*\text{Recall}}{\text{Precision}+\text{Recall}}. \end{array}$$

The other is AUC (area under ROC curve) as an evaluation indicator, which is unable to perform quantitative analysis due to the ROC curve. So, we use the area of the curve AUC (area under ROC curve) as an evaluation indicator. The AUC can be expressed by

(7) $$\begin{array}{c} \text{AUC}=1-\frac{1}{m^{+}m^{-}}\underset{x^{+}\in D^{+}}{\sum }\underset{x^{-}\in D^{-}}{\sum }\left(W\left(f\left(x^{+}\right)<f\left(x^{-}\right)\right)\right)-\frac{1}{m^{+}m^{-}}\underset{x^{+}\in D^{+}}{\sum }\underset{x^{-}\in D^{-}}{\sum }\left(\frac{1}{2}W\left(f\left(x^{+}\right)=f\left(x^{-}\right)\right)\right). \end{array}$$

In formula (7), *D*^+^ is the set of all positive samples; *x*^+^ is one of the positive samples; *D*^−^ is the set of all negative samples; *x*^−^ is one of the negative samples; *f*(*x*) is the prediction result of the model for the sample *x*, between 0 and1; and *w*(*x*) takes 1 only if *x* is true, and 0 otherwise.

### 4.2. Parameter Selection and Model Analysis

In experiments to verify the effectiveness of data preprocessing and data enhancement, the parameters such as optimization method, learning rate, and iteration number adopted are only an initial selection setting, which may not be the most suitable parameters for the model. Therefore, in order to find the optimal parameter settings, in the MFSCNet A model according to the parameters set by different experiment comparison, the results are shown in Table 3 below. When other parameters are set the same, different optimization methods are used to carry out experiments. The experimental results show that compared with stochastic gradient descent (SGD), the average accuracy obtained by Adam optimization method is higher, and the convergence speed of Adam is faster in the training process. Then, other parameters are fixed and the image size is adjusted. When the input image size is 224 × 224, the model accuracy is the highest. Then, through experimental comparison, the optimal batch size is 32, the optimal learning rate is 0.0001, and the optimal number of iterations is 500 or 1000.When the model MFSCNet C uses the optimal parameter settings, binary classification of the average accuracy rate can reach 99.48%.

The parameters of the three models proposed in this paper, MFSCNet A, MFSCNet B, and MFSCNet C, are set as the optimal parameters obtained from the above experiments, and the dichonomy and multiclass classification experiments are carried out. In the binary classification experiment, 2000 benign pathological images and 2000 malignant diseases were randomly selected from the BreakHis dataset. The selected images are randomly divided, and then, data preprocessing and data enhancement are carried out. In the multiclass classification experiment, 400 images are randomly selected from each subtype of the BreakHis dataset as the multiclass classification experimental data. The selected images are also randomly divided, and then, the data preprocessing and data enhancement are carried out. The above data are randomly divided according to the ratio of training set, verification set, and test set 7 : 1 : 2. The experimental results are shown in Table 4 below. In binary classification model, MFSCNet A accuracy is 99.05% ~99.89%, MFSCNet B accuracy is 98.06% ~99.32%, and MFSCNet C accuracy is 98.81% ~99.36%. Multiclass categories are as follows: model MFSCNet A accuracy of 94.36% ~98.41%, MFSCNet B accuracy is 91.76% ~94.05%, and MFSCNet C accuracy is 94.76% ~97.07%. Especially, the MFSCNet A network model has obtained the best performance in the high-precision classification experiments of mammary cancer. The experimental results of MFSCnet A in binary classification and multiclassification are shown in Figure 10. The change curve of the multiclass AUC value is shown in Figure 11, and it can be clearly seen that the AUC has always been a value close to 1. At the same time, the experiment was compared with DenseNet121; the results showed that the original DenseNet121 did not have a high classification accuracy for mammary pathology images. The accuracy of binary classification was 90.01% ~91.91%, and the accuracy of multiclass classification was only 79.19% ~83.30%, which was significantly lower than the proposed classification method in this paper. And according to Table 4, MFSCNet A precision rate and recall rate and other evaluation index are better than the same DenseNet121 and MFSCNet B and MFSCNet C. Especially, the MFSCNet A network model has obtained the best performance in the high-precision classification experiments of mammary cancer.

From the above experimental results, it can be seen that in this paper the mammary cancer classification model MFSCNet A by adjusting the parameters was proposed, the optimal parameter settings for MFSCNet A are obtained, and high-precision classification of mammary tissue pathological images can be performed. In this paper, MFSCNet A is used in the mammary cancer classification algorithm.

### 4.3. Ablation Experiment

To verify the effectiveness of SENet in convolutional neural networks before and after optimization, we conduct binary classification ablation experiment on the BreakHis dataset. Since the algorithm proposed in this paper mainly introduces the SENet module with optimization operations such as local pooling, global pooling, and variance directly into the DenseNet121 architecture, and we have selected the optimal network model MFSCNet A in this paper. Therefore, DenseNet121 is used as the benchmark and the optimization operation SEDenseNet121 is not introduced in SENet, and the optimization operation MFSCNet A is introduced for ablation experiment. The experimental results are shown in Table 5 below.

It can be seen from Table 5 that the performance tests of SENet before and after optimization are added to the DenseNet121 architecture in different situations. The test performance of SEDenseNet121 before adding the unoptimized operation has been improved, and the performance is improved by 6.8% compared with that of DenseNet121; the test performance of MFSCNet A is also improved after adding the optimization operation, and the performance is improved by 8.43% compared with that of DenseNet121.

### 4.4. Compare That with Other Experiments

To demonstrate the superiority of this method, we compare MFSCNet A with other mammary histopathological image classification methods for binary and multiclassification experiments. In the following experimental analysis, the datasets used by MFSCNet A and other classification methods are the breast histopathological image dataset BreakHis. The comparison results are shown in Table 6. Wei et al. [16] proposed an advanced data augmentation method and a novel mammary histopathology image classification method (BiCNN) based on the deep convolutional neural network GoogleNet. But, this method only conducts binary classification experiments of mammary cancer, and the classification accuracy is between 97.56% and 97.97%. Han and Wei [25] proposed a new class structure-based deep convolutional neural network- (CSDCNN-) based breast pathological image recognition method. The classification accuracy of the binary classification experiment is between 95.7% and 97.1%, and the accuracy of the multiclass classification experiment is between 93.2% and 94.7%. Bardou et al. [26] designed a CNN topology and used data augmentation for classification experiments. The final accuracy of the binary classification is between 96.15% and 98.33%, and the accuracy of the multiclassification experiment is between 92.8% and 93.9%. Jiang et al. [17] proposed a new learning rate scheduler. And design of a novel CNN architecture for breast histopathology image classification utilizing a small SE-ResNet module. This network is named breast histopathology image classification network (BHCNet). The final accuracy of the binary classification is between 98.87% and 99.04%, and the accuracy of the multiclassification experiment is between 90.66% and 93.74%.The above experimental results and analysis show that the overall performance of MFSCNet A is better than other methods such as BHCNet.

According to the experimental results, MFSCNet, the mammary pathology image classification model proposed in this paper, has a higher classification accuracy than the original DenseNet121 without the SE module, because it integrates the spatial and channel characteristic information. And because MFSCNet A than SE module is inserted into the DenseNet transition layer which is inserted into a dense block, therefore, MFSCNet A can turn a dense block, and transitional layer channel characteristic information fusion feature information and space, more image features are learned, which makes the performance of this network model better than the other two network models. In addition, it can be seen from Table 2 that the addition of SE module only increases a small amount of computation and does not have a great impact on the training time of the network.

The above experimental results and analysis proved that the overall performance of the proposed mammary pathological image classification model MFSCNet was superior to other methods in both the binary classification task and multiclassification task of mammary cancer pathological images. Especially, the MFSCNet A network model has obtained the best performance in the high-precision classification experiments of mammary cancer.

In binary classification and multiclass classification experiments, *F*1 score and other indicators were added into the evaluation indicators of the model. The specific comparison results are shown in Table 7.

## 5. Conclusions

In this paper, a high-precision classification model of mammary cancer MFSCNet based on improved DenseNet is designed, and a classification method of mammary cancer pathological images is proposed, which can achieve high-precision classification of mammary cancer pathological images. MFSCNet is based on the CNN model DenseNet and SENet. The SE module is used to learn the channel information of dense block and transition layer in the DenseNet model, and the learned channel feature information is fused with the spatial feature information of dense block and transition layer to realize the fusion of image space feature and channel feature.

According to insert the number and location of different SE modules, model learning channel information is different and can be divided into MFSCNet: MFSCNet A, MFSCNet B, and MFSCNet C 3 kinds. In this method, a color normalization method and different data enhancement operations are also used to deal with mammary adenocarcinoma tissue pattern image data database BreakHis. Through experiments, it is verified that data preprocessing and data enhancement processing can further avoid overfitting in the process of model training and improve classification performance. Finally, the experimental results show that the model can put forward three MFSCNet networks. MFSCNet A has obtained the best classification performance. The accuracy of dichotomous tasks ranged from 99.05% to 99.89%, and multiclass classification task identification accuracy was between 94.36% and 98.41%.

At present, we can only accurately classify the breast histopathology images in the binary classification and multiclassification experiments. It is still not possible to make an accurate detection of the lesion area. Therefore, our next work can start from detecting the lesion area of the breast histopathology images, the overlapping of cells in mammary cancer pathology images was observed by different devices, and then, the location of the target was used to mark the core location of the lesion, The computer-aided diagnosis can meet the clinical needs and is more conducive to the treatment of mammary cancer.

Moreover, through comparative analysis with other mammary histopathological image classification models, it is proved that the classification performance of MFSCNet A proposed in this paper is superior to other methods. In this paper, it has been fully proved that MFSCNet can accurately classify mammary tissue images and has great application prospects in predicting the degree of tumor.

## Figures and Tables

**Figure 1:** Classification of mammary pathological images.

**Figure 2:** An image sample of the BreakHis database. Different magnifications: (a) 40x, (b) 100x, (c) 200x, and (d) 400x.

**Figure 3:** Normalized histopathology image.

**Figure 4:** Data augmentation for different flip angle plots.

**Figure 5:** Structure diagram of the handwriting character recognition convolutional neural network.

**Figure 6:** The dense block with 5 convolutional layers.

**Figure 7:** Structure of the SE module.

**Figure 8:** Add SENet model after optimized operation.

**Figure 9:** Insertion locations for different network model SE modules.

**Figure 10:** Accuracy variation curves of MFSCNet A binary classification and multiclass classification.

**Figure 11:** Multiclass classification AUC value change curve.

**Table 1:** The specific distribution of the BreakHis dataset.

Magnification	Benign	Malignant	Combined
40x	625	1370	1995
100x	644	1437	2081
200x	623	1390	2013
400x	588	1232	1820
Total	2480	5429	7909
Patients	24	58	82

**Table 2:** The number of training parameters of different network models.

Network model	Number of training parameters (one)	
	Binary classification	Multiclass classification
ResNet18	11172866	11175944
DenseNet121	7544518	7550788
DenseNet169	13172550	13182660
DenseNet201	18887494	18899140
DenseNet264	31593926	31610180
MFSCNet A	7606190	7612460
MFSCNet B	7553914	7560184
MFSCNet C	7596794	7603064

**Table 3:** Average accuracy obtained by adjusting different parameters.

Image size	An optimization method	Vector	Batch size	The number of iterations	Average accuracy (%)
224 × 224	Adam	0.001	32	500	99.06
224 × 224	SGD	0.001	32	500	97.69
256 × 256	Adam	0.001	32	500	98.75
448 × 448	Adam	0.001	8	500	97.88
512 × 512	Adam	0.001	8	500	98.12
224 × 224	Adam	0.001	16	500	98.92
224 × 224	Adam	0.0001	32	500	99.48
224 × 224	Adam	0.0001	32	300	99.05
224 × 224	Adam	0.0001	32	1000	98.99

**Table 4:** Classification accuracy of different models for images with different magnifications.

Network model	The experimental type	Accuracy of different magnification (%)			
		40x	100x	200x	400x
DenseNet121	Binary classification	90.90	90.01	91.91	91.66
	Multiclass classification	82.24	79.19	81.23	83.30

MFSCNet A	Binary classification	**99.51**	**99.46**	**99.89**	**99.05**
	Multiclass classification	**97.13**	**94.36**	**98.41**	**95.96**

MFSCNet B	Binary classification	98.97	98.55	98.06	99.32
	Multiclass classification	93.01	93.73	94.05	91.76

MFSCNet C	Binary classification	99.36	99.05	99.00	98.81
	Multiclass classification	92.91	92.03	91.47	92.51

**Table 5:** Optimization operation.

Algorithm name	SENet without introducing optimization operations	SENet introducing optimized operations	Correct rate
DenseNet121			91.05
SEDensenet121	✓		97.85
MFSCNet A		✓	99.48

**Table 6:** Comparison of the results of binary classification experiments and multiclassification experiment with MFSCNet and other methods.

Methods	Classification task	Accuracy of different magnification (%)			
		40x	100x	200x	400x
BiCNN	Binary classification	97.89	97.64	97.56	97.97
	Multiclass classification	—	—	—	—

CSDCNN	Binary classification	97.1	95.7	96.5	95.7
	Multiclass classification	94.1	93.2	94.7	93.5

CNN	Binary classification	98.33	97.12	97.85	96.15
	Multiclass classification	92.8	93.9	93.7	92.9

BHCNet	Binary classification	98.87	99.04	99.34	98.99
	Multiclass classification	93.74	93.81	92.22	90.66

MFSCNet A	Binary classification	**99.51**	**99.46**	**99.89**	**99.05**
	Multiclass classification	**97.13**	**94.36**	**98.41**	**95.96**

**Table 7:** Comparison of evaluation results of multiclass classification methods in different classification tasks.

Methods	Classification task	Average accuracy (%)	Mean accuracy (%)	Average recall rate (%)	Average *F*1 value (%)
DenseNet121	Binary classification	91.05	91.34	92.01	91.76
	Multiclass classification	84.01	83.73	85.98	84.84

MFSCNet A	Binary classification	**99.48**	**99.61**	**99.23**	**99.42**
	Multiclass classification	**96.71**	**97.02**	**96.54**	**96.78**

MFSCNet B	Binary classification	98.73	97.34	98.84	97.65
	Multiclass classification	93.14	93.42	92.95	93.18

MFSCNet C	Binary classification	99.06	98.86	98.48	98.67
	Multiclass classification	92.23	91.34	93.18	92.25

## Data Availability

The data used to support the findings of this study are included within the article.
